# The Plausible Relationship Between Periodontitis and Glaucoma

This article has been retracted.

**DOI:** 10.7759/cureus.27440

**Published:** 2022-07-29

**Authors:** Kamakshi Gupta, Navneet Kaur, Gurpreet Kaur

**Affiliations:** 1 Department of Periodontics, National Dental College and Hospital, Derabassi, Mohali, IND; 2 Department of Periodontics and Implantology, National Dental College and Hospital, Derabassi, Mohali, IND

**Keywords:** diabetic retinopathy, uveitis, periomedicine, periodontitis, inflammation, retinal ganglion cells, glaucoma

## Abstract

Periodontitis has been associated with several medical conditions. For some of these medical conditions, periodontitis has been hypothesized to share important pathogenic mechanisms with other systemic conditions affecting the body. Recently, advances in technology have led to the identification of novel inflammatory mediators implicated in some chronic medical conditions associated with periodontitis. The potential identification of these systemic inflammatory mediators in periodontitis would offer additional support to the potential periodontal-systemic disease association. In recent years, the term oral foci of infection has attained an upturn in terms of systemic morbidities, while finite scrutinization indicates the implication of chronic oral inflammation in the pathogenesis of eye diseases. Initially, there is a singularity for the mechanistic understanding of the reported link between periodontal diseases and ocular comorbidities. There is a limited number of scientific evidence in the literature that suggests a relationship between glaucoma and periodontitis, and they share a common pathway/link based on inflammatory markers. Based on a molecular biological technique, it was believed by researchers and clinicians that eye diseases were a result of oral infections. Furthermore, this review will try to focus on the concept of oral dysbiosis in the progression of inflammatory eye diseases such as diabetic retinopathy, scleritis, uveitis, glaucoma, and age-related macular degeneration (AMD).

## Introduction and background

Periodontal disease is an inflammatory disease caused by bacterial infection of the teeth and the supporting structure of the periodontium [1]. The prevalence of periodontists in adults is over 46%; it is a major public dental health problem [2]. The potential risk factors for periodontitis are smoking, diabetes, and a number of systemic diseases that may lead to the high prevalence of periodontitis [3]. Periodontitis is associated with an era of systemic conditions and diseases such as cardiovascular diseases, diabetes, psoriasis, rheumatoid arthritis, pregnancy outcomes, and respiratory diseases. These systemic diseases have a direct or indirect relationship with periodontitis [4]. The hypothesis is that oral infections have an effect that has gone beyond the oral cavity and involves systemic diseases. This hypothesis is supported by the evidence through a number of intervention studies. Some significant publications have been compiled by the European Federation of Periodontology (EFP) and the American Academy of Periodontology (AAP) in a jointly held workshop conducted in the year 2013. In a more recent review, systemic disorders and medication that may affect the periodontal tissues and are associated with the profound loss of periodontal attachment and alveolar bone have been summarized.

In today’s era, periodontal disease is associated with dysbiosis of oral microflora. The oral cavity provides various habitats for the colonization of microflora, which may harbor the oral cavity and human aerodigestive tract. The oral cavity is the only part of the body through which microorganisms may gain access to distant body organs, and the majority of anaerobic microflora may gain access and cause infectious diseases in the body [5]. The microflora releases various endotoxins and causes the destruction of the soft tissue, which may lead to the generation of inflammatory markers such as cytokines, eicosanoids, TNF-α, and matrix metalloproteinases (MMP) that cause the disintegration of connective tissue and alveolar bone. Neutrophils play a primary role in the host response against the invading periodontopathogenic microorganisms. The presence of inflammatory mediators such as IL-β, which have a predominant role in defining different diseased states, is increased in periodontal diseases. So far, the direct effect of dysbiotic oral microbiota on systemic disease is not fully understood; however, good oral hygiene as a preventive measure is stated to be an important parameter to prevent bacterial dissemination to the other parts of the body.

In 1996, Offenbacher introduced the concept of periodontal medicine. Based on the relationship and biological plausibility through various human and animal studies, there are several studies in the literature that hypothesize that periodontal pathogens may contribute to a number of systemic diseases that may affect the oral cavity either directly or indirectly [1]. In recent days, researchers and investigators are exploring a new link between eye disease and periodontitis; however, no mechanism directly describes this association. Periodontitis still greatly impacts general health and visual function (Figure 1). The scientific gap in this association may open a new direction for analyzing the noble relationship between chronic inflammatory conditions, such as age-related macular degeneration, uveitis, diabetic retinopathy, glaucoma, and scleritis, and periodontal diseases.

**Figure 1:** Normal retina and periodontium versus retina and periodontium with diseases

## Review

Epidemiological evidence of the association between periodontal disease and eye disease

There may be a possibility that oral infection may induce eye problems, which has been demonstrated in the scientific literature. Sepić-Bilić et al. in 2008 reported that patients with inflammation associated with the hard and soft tissues of the oral cavity have central retinitis. Similarly, a significant correlation between uveitis and oral infection was also reported [6]; however, the evidence of the association between periodontal disease and eye disease is fairly recent. 

Scientific data also reported that patients with gingivitis had an increased risk (57%) of retinal hemorrhage. Recent data on this subject suggested that there is a link between periodontal disease and age-related macular degeneration, which is one of the important causes of irreversible central vision loss in older people more than the age group of 60 years. Astafurov et al. in 2014 conducted a pilot case-control study and stated that peripheral and extraocular bacterial activity could be potentially contributed to the pathogenesis of glaucoma. In this study, mouthwash specimens with test patients with glaucoma and control subjects were analyzed for bacterial load volume [7]. The oral bacterial load in patients with glaucoma was significantly higher than those patients without glaucoma, which may suggest that glaucoma patients may be constantly exposed to a higher level of bacterial products and may exacerbate the severity and disease progression [8].

In 2019, Azam et al. stressed the upregulation of the complement system and Toll-like receptor-4 (TLR4) signaling activity in the pathological tissue along with microglial cell activation, which is associated with the optic nerve and plays an important role in neurodegeneration. Toll-like receptors (TLRs) are predominantly involved in the pathogenesis of many neurodegenerative eye diseases, including glaucoma [9]. A pilot study conducted by Polla et al. in 2017 suggested that no variation in the volume of oral bacterial load may be directly linked with glaucoma pathology. The results of this case-control study revealed that there was a higher number of streptococci in open-angle glaucoma cases as compared to control cases. Moreover, scientific evidence indicated that the existence of the relationship between periodontal disease and eye disease such as glaucoma is based on the increased production of inflammatory markers such as IL-6, IL-8, and TNF-α and the activation of several complement fragments (C3a, C5a, and C4a) in host immune response [10].

Innate immune system: a key marker bridge between periodontal disease and glaucoma

Glaucoma is defined as multifactorial chronic progressive optic neuropathy caused by a group of ocular conditions that may cause a progressive loss of retinal ganglionic cells and their axons, followed by a gradual loss in the visual field, which may lead to blindness. Glaucoma is the second most common cause of blindness worldwide and was estimated to affect 79.6 million people worldwide by 2021 [11]. There are various risk factors for glaucoma, ranging from age to family history, to diabetes, to hypertension, as well as other eye diseases such as high myopia. The secondary etiological factors are trauma, inflammation, and certain medication such as corticosteroids. The elevation in the intraocular pressure is the main diagnostic marker and the only modifiable risk factor for glaucoma. However, glaucoma can occur with normal intraocular pressure, which is in the range of 10-21 mmHg.

According to the International Society of Geographical and Epidemiological Ophthalmology (ISGEO), glaucoma is classified into two main groups: primary adult glaucoma, which consists of two separate conditions, open-angle and angle-closure glaucoma, and secondary glaucoma, which is due to a specific anomaly or disease of the eye (congenital or developmental glaucoma). Primary open-angle glaucoma (POAG) is a chronic, ischemic, progressive optic neuropathy that most commonly occurred in adults; it is characterized by accelerated ganglionic cell death and subsequently axonal loss. There is a progressive glaucomatous optic disc changes, glaucomatous optic disc atrophy, and corresponding loss of visual field. The intraocular pressure is raised to more than 21 mmHg, which allowed an open anterior chamber angle on gonioscopy (Figure 2). The visual field is also affected, which may present evidence of glaucomatous optic nerve head damage on fundus examination.

**Figure 2:** Pathophysiology of glaucomatous optic nerve damage

Based on clinical signs and symptoms, researchers have hypothesized that chronic subclinical peripheral inflammation induced by the non-ocular microbiome may contribute to neurodegeneration in glaucoma. Moreover, microbial dysbiosis has also been related to a number of epigenetic changes such as a significant upregulation and downregulation of histone deacetylase 2 and 3 and H4 expressions, respectively, in retinal ganglionic cells.

The most common form of glaucoma in many countries is primary open-angle glaucoma; it accounts for 60%-70% of cases in the United States. Worldwide, over two million people develop this condition every year. The most recent US study estimated that the overall prevalence rate of primary open-angle glaucoma is 1.9% in the age group above 40 years with Black people having three times more prevalence than White people [12].

Innate immunity key marker

Innate immunity has been suggested to play a significant role in chronic inflammatory disease in periodontitis. Periodontal pathogens may induce a local inflammatory response and activate innate immunity through the activation of Toll-like receptors (TLRs), which may result in the production of pro-inflammatory cytokines and the recruitment of phagocytes and lymphocytes into the inflammatory zones [13]. Simultaneously, in the retinal immune system, retinal pigment epithelium cells may play a significant role in immune response and express Toll-like receptors along with a rich source of pro-inflammatory cytokines, chemokines, and growth factors (Figure 3) [14,15]. The complement system is the backbone of the innate immune system. The activation of the complement system may produce many complement fragments such as C3a, C4a, and C5a in ocular disorders and periodontitis. Therefore, complement dysfunction plays an important role in periodontitis and eye diseases and could be a common pathway to establishing a strong relationship between these two diseases [16].

There is genetic polymorphism in the genes encoding the complement pathway. Fragment C5 is associated with an increased risk of acute anterior uveitis in the Chinese population [17]. Moreover, preclinical and clinical studies have suggested the primary role of the complement pathway in acute macular degeneration pathophysiology [18]. A similar type of scientific evidence in the literature has highlighted the clinical implication of the complement pathway in the pathogenesis of periodontal diseases [19]. In the case of induced gingivitis, there is an increased proportion of C3 complement cleavage in the gingival crevicular fluid (GCF). Moreover, if periodontal treatment is given to such cases, it may lead to the reduction of the C3 complement cleavage rate in human GCF [20]. In preclinical study models, the use of complement inhibitors for the treatment of periodontal disease has been recently demonstrated, and these models highlighted the positive and beneficial effects on the treatment of periodontal diseases. Alteration in the complement pathway and innate immunity key marker form a bridge to establish a relationship between periodontitis and eye diseases such as glaucoma [20].

Generally, the ocular immune system provides protection to our eyes from external and internal stimuli and enhances the healing processes. The blood-retina barrier, immune status of the retina, microglial cells, and complement defense system help maintain retinal homeostasis. It also prevents the trafficking of the cells and large molecules to and from the eyes. Under certain conditions such as infection and trauma, there is a breakdown in the blood-retina barrier along with impairment in the retinal pigment epithelium, which may result in the direct or indirect impairment of retinal neurons during the inflammatory conditions in both diseases. Periodontal pathogens (red, orange, yellow, green, and purple complex), immune cells (lymphocytes, monocytes, natural killer cells, and Th 17), and altered levels of inflammatory mediators (IL-1, IL-6, TNF-α, PGE2, and C-reactive protein) are responsible for periodontal diseases and eye diseases such as glaucoma, diabetic retinopathy, uveitis, and age-related macular degeneration (Figure 3). Scientific evidence in the literature suggests that local or systemic inflammation along with alteration in the inflammatory pathway is most likely a key link between periodontal diseases and eye diseases.

**Figure 3:** Involvement of oral pathogens, immune cells, and altered levels of inflammatory mediators in different eye diseases NK: natural killer cells; MØs: macrophages; IICs: inflammatory immune cells; IL: interleukins; TNF-α: tumor necrosis factor-alpha; TGF-β: transforming growth factor-beta; CRP: C-reactive protein

## Conclusions

The mechanism of the relationship between periodontitis and glaucoma is not clear. However, several scientific studies in the literature have reported the association between periodontal diseases and glaucoma. Moreover, certain hypotheses suggest that there is a potential association of innate immunity involvement with similar risk factors for both diseases. Periodontal diseases may also be considered an additional risk factor for having eye diseases such as glaucoma, uveitis, diabetic retinopathy, and age-related macular degeneration. More evidence-based scientific research is needed to confirm this existence, whether this would be unidirectional or bidirectional or could be a common thread that links eye diseases and periodontitis. Therefore, further interventional and epidemiological studies would be necessary to provide a better understanding of this type of association.
